The article "Research on Image Segmentation Algorithm Based on Multimodal Hierarchical Attention Mechanism and Genetic Neural Network" was published in 2022. Journal: Comput Intell Neurosci.

# Research on Image Segmentation Algorithm Based on Multimodal Hierarchical Attention Mechanism and Genetic Neural Network

**DOI:** 10.1155/2022/9980928

**Published:** 2022-06-06

**Authors:** Dalei Wang, Lan Ma

**Affiliations:** ^1^School of Mechanical and Electronic Engineering, Suzhou University, Suzhou, Anhui 23400, China; ^2^School of Math and Statistic, Suzhou University, Suzhou, Anhui 23400, China

## Abstract

Multimodal tasks based on attention mechanism and language face numerous problems. Based on multimodal hierarchical attention mechanism and genetic neural network, this paper studies the application of image segmentation algorithm in data completion and 3D scene reconstruction. The algorithm refers to the process of concentrating attention that humans subjectively pay attention to and calculates the difference between each pixel in the genetic neural network test image in the color space and the average value of the target image, which solves the problem of static feature maps and dynamic feature maps of image sequences. In addition, in view of the problem that the number of attention enhancement feature extraction modules is too large and the parameters are too large, the recursive mechanism is used as the feature extraction branch, and new model parameters are not added when the network depth is increased. The simulation results show that the accuracy of the improved image saliency detection algorithm based on the attention mechanism reaches 89.7%, and the difference between the average value of the single-point pixel and the target image is reduced to 0.132, which further promotes the practicability and reliability of the image segmentation model.

## 1. Introduction

In recent years, neural network technology has developed rapidly, and image segmentation technology has also developed more and more mature, and the application field of image segmentation has become more and more extensive [1]. Image segmentation is a relatively popular subresearch direction in the general field of genetic neural network machine attention mechanism. Image segmentation technology can segment some target objects in specific modes by extracting and understanding image features. At present, there are many research applications of image segmentation technology, such as face segmentation, license plate segmentation, commodity segmentation, fingerprint segmentation. Attention mechanism has three main functions in attention mechanism question answering: first, the mechanism can locate and extract effective information according to the specific questions asked; second, the attention mechanism can semantically align the natural language and the attention mechanism pictures, so as to realize inference at a more fine-grained level to increase the interpretability of the model [2–5].

The article "Research on Image Segmentation Algorithm Based on Multimodal Hierarchical Attention Mechanism and Genetic Neural Network" was published in 2022. Journal: Comput Intell Neurosci.

In the analysis, understanding and processing of images or image resources, researching and improving the saliency detection algorithm of images can not only filter out important information in the analysis and processing work but also can obtain relatively fast results in the analysis and problem-solving. In the subsequent work of image editing or adaptive compression, resources can be reasonably allocated to reduce the damage to resource information during image transmission and processing [6–8]. It may try to use a method based on the adversarial complementary attention mechanism, which can not only extract the main salient discriminative features of the image but also the secondary salient discriminative features of the image. This method mainly includes two classifiers, where Classifier A is used to learn some particularly significant discriminative features of objects. Classifier B erases these discriminative features learned by classifier A, and then learns the next discriminative feature, that is, compared with classifier A. The experimental results show that this genetic neural network image segmentation method based on adversarial complementary attention can improve the accuracy of genetic neural network image segmentation. On the one hand, the high-level semantics generated from images can narrow the semantic gap between the attention mechanism of images and natural language questions, enabling reasoning in a common semantic space; on the other hand, compared with traditional image features, high-level semantics are readable and interpretable and thus provide a basis for reasoning about answers and diagnosing errors in question answering systems. However, existing automatic attention mechanism question answering models usually have the following two problems [9–11].

To solve this problem, this paper proposes a multimodal hierarchical estimation model based on multimodal hierarchical neural network and multimodal input, and obtains reliable multimodal hierarchical regions by combining traditional methods (stereo matching, hardware sensors, etc.), to recover a more accurate and dense multimodal level estimation result. The model takes RGB images and sparse but reliable multimodal hierarchical sampling as input, extracts effective information from the input through the method of adversarial learning, and models the multimodal level of the scene to achieve traditional methods and deep neural-based methods. The advantages and disadvantages of the network monocular prediction method are complementary to achieve better multimodal level restoration results. First, the questions asked by the automatic attention mechanism are diverse and complex. Existing works usually use a single-level image representation, which cannot meet the information required by various questions. Second, the existing attention models independently inherit different regions of the image. The neural network attention weight ignores the contextual information between objects in the image and cannot answer questions that require relational reasoning. Based on these problems, this paper conducts in-depth research on the attention mechanism in automatic attention mechanism question answering, applies the attention network innovatively to the expression of images at different levels, and then performs more effective information extraction, understanding, and reasoning according to the questions raised. Specifically, the proposed multimodal hierarchy recovery model is divided into two main parts: the initial multimodal hierarchy estimation part and the multimodal hierarchy refinement part, which realizes the scene multimodal hierarchy estimation in a coarse-to-fine manner. The multimodal level refinement part innovatively adopts the scale residual learning method, which greatly improves the performance of the system. In addition, in order to eliminate the influence of multimodal level acquisition noise in the training data on the system training, this paper proposes a sparse discriminant network, which makes the network training process more stable and the prediction results more reliable.

The article "Research on Image Segmentation Algorithm Based on Multimodal Hierarchical Attention Mechanism and Genetic Neural Network" was published in 2022. Journal: Comput Intell Neurosci.

## 2. Related Work

Multimodal level restoration is a classic problem in the field of machine attention mechanisms in genetic neural networks. In recent years, single-view depth restoration based on multimodal hierarchical neural networks has received extensive attention in the academic community. However, the single-view multimodal hierarchical restoration based on the multimodal hierarchical neural network can often only generate fuzzy estimation results and cannot restore an accurate and consistent scene scale due to its inherent ill-posedness. According to the characteristics of the image, a specific area of the image is selected, and through rapid eye movement scanning, the area is moved to the fovea area with high resolution and attention to this area is realized for more detailed observation and analyze. The selective attention mechanism is a key technology for humans to select specific regions of interest from a large amount of information input from the outside world [12–14].

Both multigranularity curve trends and time dependencies of time series are important information useful for TSC tasks. Alhnaity et al. [15] proposed a multimodal neural network consisting of a multiscale FCN module and an LSTM module. The network also pays attention to the multiscale geometric spatial characteristics and numerical time-dependent characteristics presented by the time series curve. With a comprehensive grasp of their characteristics, the categories of the series can be better distinguished. In the model, a large-scale receptive field is achieved through the segmentation of hollow images, so as to ensure that the training pressure will not increase significantly. A series of experiments on the UCR dataset validate the effectiveness and superiority of the model. Arya and Saha [16] believes that it is only an algorithm based on histogram comparison and does not involve the content of image segmentation. Therefore, its running efficiency is faster than that of the Rc algorithm, so its real-time performance is very good. Of course, the accuracy of the saliency map generated by this algorithm will be lower than that of the Rc algorithm. In addition, since the algorithm is only a genetic neural network based on color features and does not process the multimodal hierarchical features, the algorithm cannot segment the multimodal hierarchical information in the image, and the accuracy of the saliency map rate has a big impact. Obviously, the algorithm has a very good effect on those images with strong color information and weak multimodal level information, and the LC algorithm has a very good effect on those images that are difficult to be automatically segmented.

The article "Research on Image Segmentation Algorithm Based on Multimodal Hierarchical Attention Mechanism and Genetic Neural Network" was published in 2022. Journal: Comput Intell Neurosci.

The classification method based on distance metric relies on the distance between the samples to be classified as the information on which the classification task is based. The distance may be a global distance or a local distance, and the use of distance information can be directly used as a similarity measure. At present, Manica et al. [17] believes that the research on distance-based TSC methods mainly focuses on the optimization of distance metric methods and the innovation of distance information utilization, while the classifiers used are relatively conventional, such as k-NN, SVM. Algorithms, such as decision trees, Bayes, are rarely innovative in terms of classifiers, because they are not the key to improving the performance of such methods. Yan and Zhang [18] analyzed that the two basic modules focus on feature extraction and complex function relationship fitting, respectively, and they can achieve a better state after independent training. In addition to the conventional validity verification experiments, the method has also been tried to solve the problem of aero-engine fault diagnosis in the field of traditional sequence classification, and good results have been achieved. Rafi and Das [19] proposed a locally weighted dynamic time warping algorithm LW-DTW, which can make up for the limitation of standard DTW in the classification of complex time series due to the assumption of uniform distribution of time series. There are also many solutions to alleviate the problem of ill-conditioned alignment by imposing strict constraints on the regular path, such as weighting, penalty function constraints, improved step-size increasing modes, etc. The above methods make up for the defects of DTW to a certain extent, but the overall accuracy level is still not high [20–25].

The article "Research on Image Segmentation Algorithm Based on Multimodal Hierarchical Attention Mechanism and Genetic Neural Network" was published in 2022. Journal: Comput Intell Neurosci.

## 3. Multimodal Hierarchical Attention Mechanism Network

### 3.1. Multimodal Hierarchical Topology

An elastic resource management system based on multimodal neural network can be used to solve the above problems. The system includes an initial resource recommendation module and an elastic resource management module. The initial resource recommendation module will recommend the genetic neural network resource configuration that can complete the task on time and the least rental cost for the tenant according to the deadline and workload of the tenant's genetic neural network task.

During the genetic neural network process of the task, the multimodal neural network of the elastic resource management module can extract the characteristics of three modalities, such as the number of genetic neural network resources, the utilization rate of genetic neural network resources, and the speed of the task genetic neural network, and analyze the task in real time. This prediction model can timely capture the changes in the speed of the task genetic neural network and adjust the prediction results when the performance of the virtual machine is degraded. When it is predicted that the completion time of the genetic neural network task exceeds the deadline, the system will increase the number of genetic neural network resources, improve the genetic neural network speed of the task, and finally ensure that the task is completed on time:

(1) $$\begin{array}{c} K\left(e,e{}^{\prime }\right)=E\left(i,j\right)\times \left|e\left(\text{cos}t,\text{sin}t\right)-e{}^{\prime }\left(\text{cos}t,\text{sin}t\right)\right|. \end{array}$$

Finding the object in the most discriminative area of the image, erase the area from the image, and then retrain the classification neural network to find another area of the object, and so on, iteratively learn until the trained neural network is in it, and these regions are combined to form a new discriminative region for semantic segmentation. The specific erasing method is to set the value of the corresponding pixel point to the average value of all training set image pixels. Saliency feature extraction has great application value in image retrieval, authentication, segmentation, matching, and other research fields. Introducing this perception-based selection mechanism into the field of image analysis and prioritizing genetic neural network resources to those areas that are easy to attract the attention of the observer will greatly improve the efficiency of existing image analysis methods. When designing an image retrieval or Hash algorithm, it is obviously not feasible to manually point out the area that attracts attention for each image and then focus on extracting the features of this area:

(2) $$\begin{array}{c} \text{for}\left\{\alpha \left(i,j\right),i,j\rangle 0\right\},\text{max}\left\{\frac{\text{d}\alpha }{\text{d}t}+\frac{\text{d}\alpha }{\text{d}j}+\frac{\text{d}\alpha }{\text{d}i}\right\}\rangle 1. \end{array}$$

Multimodal hierarchical feature is another important feature of low-level attention mechanism of image. Its essence is to describe the spatial distribution of grayscale in the neighborhood of pixels. Multimodal hierarchy primitives are the basic elements that make up a multimodal hierarchy. The proposed color moments (moments) are very simple, and the effective methods for color feature are extraction and matching. Any color distribution in an image can be represented by its moments. Here, the color distribution of the image can be roughly expressed by using only the first, second, and third moments of the color, because most of the color distribution information is concentrated in the low-order moments. It does not require vectorization of color features which is another advantage over color histograms. Therefore, the color moment of the image only needs a total of nine components (three color components, three low-order moments on each component), which is more concise than other color features. Color moments are often used in combination with other features as prefiltering to narrow the scope of the study, that is, for the initial inspection of image retrieval.

The article "Research on Image Segmentation Algorithm Based on Multimodal Hierarchical Attention Mechanism and Genetic Neural Network" was published in 2022. Journal: Comput Intell Neurosci.

### 3.2. Image Neural Network Node Distribution

Receptor cells can convert light quantum energy into electrical signals. Specifically, light stimulation becomes the hyperpolarization of the membrane potential of the sensor cells, and the signals are transmitted to bipolar cells through chemical synapses, which in turn process the signals. The decoder uses the attention mechanism to perform beam search decoding and takes the text as the output and calculates the context vector at the current moment through the attention model to more accurately output the text description that matches the speech.

(3) $$\begin{array}{c} \sum_{y,k}^{y+k}\left(\frac{\text{d}\alpha }{\text{d}t}+\frac{\text{d}\alpha }{\text{d}j}+\frac{\text{d}\alpha }{\text{d}i}\right)-\sum_{y,k}^{y-k}\left(\frac{\text{d}\beta }{\text{d}t}+\frac{\text{d}\beta }{\text{d}j}+\frac{\text{d}\beta }{\text{d}i}\right)=0. \end{array}$$

The spatial directional relationship is described by the directional relationship diagram. Two objects are connected by an edge in the relational graph, and the slope of the connection corresponding to the fixed point is represented by the weight on the edge. The edge table describing the object is composed of a set of all edges, and the edges are arranged according to the lexicographical order of the symbols. The similarity between spatial layouts is described by the similarity of orientation graphs. Object modeling and segmentation are the core issues of object semantic content acquisition. The spatial relationship between objects is to further describe the relationship between the objects after they are segmented. This can obtain the internal representation of the objects through data mining and machine learning methods, and the classification of objects requires pattern segmentation.

In the IT model, a Gaussian filter is used to gradually linearly filter the input image in Figure 1, and the input image is gradually sampled from the horizontal and vertical directions to obtain nine images of different sizes. The filtered and sampled images are distributed in the 0th–8th layers of the Gaussian pyramid, where the 0th layer image is sampled at 1 : 1, that is, the original image size is preserved, and the 8th layer is sampled at 1 : 256. Then, the chromaticity (colors) features, the intensity features, and the orientation features are extracted for each layer of the image in the pyramid. Afterwards, by simulating the antagonistic structure of the “center-week-week” of the biological receptive field, a rough feature map is obtained after normalizing the difference of the “center-week-week” of the neural network. The “center-periphery” difference (predefined by denoting O) refers to the difference between the antagonism of a single-point pixel between the “center” fine dimension c and the “periphery” coarse dimension S:

(4) $$\begin{array}{c} f\left(x,x{}^{\prime },y,y{}^{\prime }\right)=\left\{\begin{array}{cc} \left|\text{delta}\left(x,x{}^{\prime }\right)-\text{delta}\left(y,y{}^{\prime }\right)\right|, & x\langle y\\ 1, & \text{otherwise}. \end{array}\right. \end{array}$$

In image retrieval, the position of objects in the image and the spatial relationship between the objects are also important features, and different images can be distinguished by understanding the spatial relationship between the objects in the image. The relationship between spatial objects with spatial characteristics is the spatial relationship, which mainly includes three categories: measurement, direction, and topology. The most direct representation is the Cartesian coordinate system, for example, a blue sky and a blue ocean are very distinguishable due to the closeness of the color histograms. The spatial autocorrelation function is the similarity between a pixel in the genetic neural network window and another pixel that deviates from it by a certain spatial distance. The periodicity of the autocorrelation function reflects the recurring periodicity of the multimodal hierarchical primitives, and its decline rate reflects the thickness of the multimodal hierarchical primitives: if the multimodal hierarchy is fine, it will decrease rapidly; if the multimodal hierarchy is rough, the decline slowly. The autocorrelation function according to the multimodal hierarchy has peaks and valleys, which can be used to detect the arrangement of the primitives in the multimodal hierarchy.

The article "Research on Image Segmentation Algorithm Based on Multimodal Hierarchical Attention Mechanism and Genetic Neural Network" was published in 2022. Journal: Comput Intell Neurosci.

### 3.3. Feature Extraction of Attention Mechanism

The multimodal level restoration based on traditional attention mechanism methods or hardware devices can obtain relatively accurate results in ideal environments or ideal regions, but the effectiveness of the algorithm in nonideal regions cannot be guaranteed. Although the monocular multimodal hierarchical restoration method based on multimodal hierarchical learning can obtain relatively robust relatively multimodal hierarchical results in the local area, it cannot obtain accurate scale information due to its own ill-posedness. It is difficult to obtain accurate multimodal level restoration. Most of the existing single-view multimodal hierarchical estimation methods based on multimodal hierarchical neural networks are only based on a single-color image:

(5) $$\begin{array}{c} \max\left\{\frac{M{}^{\prime }\left(t\left(1\right)\right)\times M{}^{\prime \prime }\left(t\left(1\right)\right)}{M{}^{\prime }t\left(i\right)},\frac{M{}^{\prime }\left(s\left(1\right)\right)\times M{}^{\prime \prime }\left(s\left(1\right)\right)}{M{}^{\prime }s\left(i\right)}\right\}=\text{max}\left\{\frac{\text{log}\left(s,t\right)}{m\left(s,t\right)}\right\}. \end{array}$$

As the network input, a function *f* is learned by training a large number of color images and corresponding multimodal hierarchical image pairs, estimating the multi-modal hierarchy of the scene. In the 500 seconds before the operation slowed down, the predictions from mode 1 were very accurate and fit well with the ideal predictions. However, the predictions from Mode 2 are far beyond the ideal predictions and have been fluctuating wildly. This is because it takes a certain time for the running speed characteristics to reach a stable state, and the prediction results obtained before that may have large errors. However, when the performance of the virtual machine decreases, the prediction in Mode 1 cannot perceive this change, and adjust the predicted value to the ideal predicted value in time. This feature will make the system based on Modal 1 unable to perform expansion operations:

(6) $$\begin{array}{c} \int \int \sqrt{\text{log}\left(t-t^{2}-1\right)}df\;dt+\sqrt{g\left(t-t^{2}\right)}dg\;dt=1. \end{array}$$

To study the image segmentation of genetic neural network under weak supervision, it is necessary to extract the subtle discriminative features of the image. Some commonly used methods are to directly use the image segmentation neural network or the method based on the attention mechanism to extract the discriminative features of the image. This feature fusion mechanism captures more complex and higher-order relationships between self-attention features and high-level features, and obtains rich semantic information to enhance the diversity of features. Therefore, from the point of view of information theory, information can be divided into redundant parts and changing parts, and the human attention mechanism system is more sensitive to the changing parts of information. Biological attention mechanism systems tend to suppress responses to conventional (or frequently occurring) features, while remaining sensitive to unconventional features. Accordingly, the image information in Table 1 can be divided into the following two parts.

The article "Research on Image Segmentation Algorithm Based on Multimodal Hierarchical Attention Mechanism and Genetic Neural Network" was published in 2022. Journal: Comput Intell Neurosci.

The purpose of the genetic neural network saliency map is to detect the “eye-catching” area or salient area in the image, generally in the visual field, according to the spatial distribution of different features, to detect the significant local area. In order to better fuse feature maps of different scales, the model proposes a normalization function *N*(*x*). In the normalization function *N*(*o*), first, for multiple feature maps of the same feature, the salient values of single-point pixels are normalized to the region N[o], so as to eliminate the huge difference between different scales. Second, find the global maximum value M in all feature maps and genetic neural network to obtain the average value of other local maxima. Finally, through (M– and) 2 genetic neural network global saliency map. The IT model employs a simple low-level attention mechanism feature to detect salient regions in images. The regions with significant attention mechanism in the image can be detected more accurately. The IT model is the most influential computational model in the field of image saliency detection. The detection result of the IT model is relatively fuzzy, the boundary between the salient area and the nonsalient area is relatively ambiguous, and the genetic neural network takes a long time, which has strict requirements on the size of the image.

The article "Research on Image Segmentation Algorithm Based on Multimodal Hierarchical Attention Mechanism and Genetic Neural Network" was published in 2022. Journal: Comput Intell Neurosci.

### 3.4. Multimodal Data Extraction

The implementation of this system is based on the EMR service provided by Alibaba Cloud. In this system, the maximum size of the genetic neural network cluster is 40 virtual machines. Each virtual machine is equipped with a 4-core Intel Xeon E5-2682 v4 2.5 GHz CPU. The MapReduce genetic neural network task performed on the virtual machine is based on the Hadoop 2.7.2 genetic neural network framework. The programming language to implement this system is Python 3.5, and the programming framework of the neural network is TensorFlow from Google. The implementation of the initial resource recommendation module is based on the regression model introduced earlier. After the tenant has given a new computing task total amount and deadline, the initial resource recommendation module will traverse all resource allocation schemes and calculate the task completion time corresponding to these schemes. If the completion time is within the deadline, the proposal will be recorded. The model is a network whose encoder-decoder structure is both RNN. The input words are linked with the predicted translation words through the attention matrix and the alignment matrix of the input and output is obtained:

(7) $$\begin{array}{c} \text{log}\left\{\int \int \frac{n!}{r!\left(n-r\right)!}dn\;dr\right\}=f\left(\log\left(1-f\left(s,t,r\right)\right)\right)df\;. \end{array}$$

At the beginning of training, the true sample distribution generates the sample distribution and the discriminator model corresponds to the black line, green line, and blue line, respectively. It can be seen from the way that at the beginning of training, the discriminant model cannot distinguish the real samples from the generated samples well, but as the training progresses (alternately update the parameters of the discriminative model and the generative model to gradually optimize the model), the generative model image distribution gets closer and closer to the real image distribution until the final model converges. The paper shows the original images of the 10th, 20th, 30th, 40th, 50^th^, and 60th image sequence, as well as the corresponding saliency maps obtained by the experimental algorithm. The results of the comparison of the prediction effects of the multimodal neural network and the single-modal neural network are shown in the text. Among them, the coordinates on the right are the percentage of task completion of the entire genetic neural network, and the corresponding curve shows the specific status of the task completion progress. When the task running speed becomes slower, the slope of this curve will become lower. In this case, the genetic neural network slowed down at about 500 seconds for the genetic neural network task.

The article "Research on Image Segmentation Algorithm Based on Multimodal Hierarchical Attention Mechanism and Genetic Neural Network" was published in 2022. Journal: Comput Intell Neurosci.

Among them, the first line is the input image of the original image sequence, and the second line is the final saliency map of the sequence in Figure 2 obtained after fusing the static striking feature map and the dynamic striking feature map. It can be seen that the boundary of the saliency area in the saliency map is relatively blurred, but basically, it can accurately indicate the location of the salient target. In order to further distinguish the difference between significant pixels and nonsignificant pixels, we multiply the saliency values of the corresponding pixels in the static feature map and the dynamic feature map, and then normalize them to the [0, 255] interval to get the final image saliency map. The system collects a large amount of initial data through 300 runs of the above three different tasks, which are mainly derived from (1) using the monitoring system to collect resource usage data; (2) running from the Hadoop genetic neural network framework obtained from the log; (3) the resource data used by each task to run from the cloud platform bill. Among them, the genetic neural network resources used for these running tasks are randomly selected within a certain range when selecting to simulate the situation encountered by tenants in the actual genetic neural network process. These datasets are sampled through a 5-second sampling window, resulting in a standard training dataset of 30,000 sets. Among them, 80% of the data will be used for model training, and the remaining 20% will be used to evaluate the quality of the model. This setting is a common way of processing time series:

(8) $$\begin{array}{c} \langle \begin{array}{c} f\left(d,t\right)=\frac{n}{r!\left(n-r\right)!}\\ \text{sigma}\left(d,t\right)=f\left(d,t\right)\times \frac{n!}{r!\left(n-r\right)!} \end{array}. \end{array}$$

The representative image selection is to select the most representative image from the image set with the same or similar text labels to represent the entire image set so that the user can effectively understand the content of the entire image set through the representative image. Selecting representative images are generally to select several images in the image set that can represent the important information of the whole image set. Generally speaking, the image set used to select representative images contains a large number of images, and the computational complexity of the process of extracting features for each image and the analysis and processing after feature extraction will be very large. Therefore, if the saliency detection of the images is carried out in advance before the work of selecting representative images starts, the processing work is arranged in the saliency area of the image, and the interference of irrelevant backgrounds in each image is reduced, then, it can also improve the accuracy of selecting representative images.

The article "Research on Image Segmentation Algorithm Based on Multimodal Hierarchical Attention Mechanism and Genetic Neural Network" was published in 2022. Journal: Comput Intell Neurosci.

## 4. Construction of Image Segmentation Model Based on Multimodal Hierarchical Attention Mechanism and Genetic Neural Network

### 4.1. Multimodal Hierarchical Feature Coding

The multimodal dataset provides sensor movement trajectories in the form of text files, including camera translation and rotation. Each line in the text file contains a separate description of the camera pose, including the timestamp of each record and the camera pose parameters. The camera pose uses three floating-point numbers to represent the position of the optical center of the RGB camera defined by the motion capture system relative to the world origin and uses a quaternion to represent the orientation of the RGB camera optical center relative to the world origin. A self-attention mechanism is described as mapping a request Q and a series of key values K to an output value V, first computing the dot product of all keys divided by the root of the k dimensional key, and then using the softmax function to compute the output value the weight of.

The effect of the saliency map with 5 × 5 Gaussian kernel and 3 × 3 Gaussian kernel is similar, and it can generally be selected according to specific requirements in practical applications. Considering the different distribution of saliency values in single-frame image sequence images, we can adopt an adaptive segmentation threshold, that is, define its adaptive segmentation threshold as a multiple of the average value of pixels in the saliency map. Since there are many black pixels in the video saliency map, the pixels whose gray value is 0 are not considered in the pixel mean in the saliency map of the genetic neural network. According to experience, for an image with a width shape and a height day, there are hum pixels with a gray value of 0, and the adaptive threshold is taken:

(9) $$\begin{array}{c} \left[\begin{array}{cc} r!\left(n-r\right)! & -1\\ -1 & r! \end{array}\right]+\left[\begin{array}{cc} \left(n-r\right)! & -1\\ -r! & r! \end{array}\right]=\left[\begin{array}{cc} 1 & 0\\ 0 & -1 \end{array}\right]. \end{array}$$

The first row is the result of the representative image selection without the saliency detection algorithm of the image, and the second row is the result of the representative image selection with the saliency detection algorithm of the image introduced. The multiple images on the left side of the arrow in the figure represent the content of each cluster center, which is used to represent the content contained in the entire online album set, and the several images on the right side of the arrow in the figure are the representative images finally selected. It can be clearly seen from the comparison that after introducing the image saliency detection algorithm, the selected representative images more completely and comprehensively express the different contents contained in the image set. The algorithm is a focused attention process that refers to the subjective attention of the creature. The algorithm sets the evaluation criteria of salient pixels through the target image selected by the user and then selects features based on the biological attention mechanism and uses global comparison to inherit the neural network saliency map. Thereby, significant regions that are more in line with the user's subjective selection are screened out so that the image resources can be further screened.

The article "Research on Image Segmentation Algorithm Based on Multimodal Hierarchical Attention Mechanism and Genetic Neural Network" was published in 2022. Journal: Comput Intell Neurosci.

Background subtraction is an effective method for detecting motion information. Its basic idea is to use the background information in the sequence images of Figure 3 to establish a parameter model to detect the changing motion information. Generally, the current frame information of the test is compared with the established background template. The information is scored and compared to detect motion information in the image sequence. The background subtraction method must first establish a background template, and the background template needs to be able to update in real time with the change of lighting or external environment. In this model, in order to fuse the features of multiscale input images, the attention mechanism is used to calculate the weights of each scale feature extracted by the convolution layer, and then the multi-scale feature information is fused according to the weights.

The time interval between two adjacent frames is very short, and the difference between the previous frame image and the current frame image of the genetic neural network has good real-time performance. LSTM can extract information on a larger time scale, so after LSTM processing, the measurement error of the feature will be smaller than the measurement error at a certain time point. Because at a certain point in time, a sudden drop in computing speed does not necessarily mean that the performance of the virtual machine has deteriorated. But if this happens over a period of time, it may indicate a change in virtual machine performance. The memory unit in LSTM can be judged by the features of time series, and the correct information can be extracted to a higher level and passed to the neural network of the next layer:

(10) $$\begin{array}{c} \text{lim}\left\{\delta \left(x,t\right)+\delta \left(x,t-1\right)+\delta \left(x,t+1\right)\right\}=L_{\text{ground}}^{x}\left(g\left(x\right),g\left(x-1\right)\right). \end{array}$$

It can be seen from the experimental comparison that although several data-driven algorithms detect the position of the image in both images, the saliency of the red image detected by several algorithms is higher than that of the white image; however, when users focus on white images subjectively, the saliency of white images detected by the TD algorithm is much greater than that of red images. The target-driven saliency detection algorithm designed in this section is based on the target image and assigns each pixel a subjective saliency value. This paper first extracts attributes and descriptive sentences as high-level semantic interpretations of pictures, and then the inference module infers the answers by exploiting these interpretations instead of the pictures themselves.

The article "Research on Image Segmentation Algorithm Based on Multimodal Hierarchical Attention Mechanism and Genetic Neural Network" was published in 2022. Journal: Comput Intell Neurosci.

The network extracts salient features at different levels by cascading several attention-enhancing feature extraction modules. The designed attention-enhanced feature extraction module consists of recursive feature extraction branch and attention extraction branch. This paper demonstrates experimentally that such a decomposition system achieves comparable performance to baseline models, while being interpretable and capable of improving the overall system with better quality attributes and captions.

### 4.2. Genetic Neural Network Output

The saliency map extraction algorithm based on the comparison of the histogram of the genetic neural network uses color statistics for each pixel of the input image to define the saliency value. The saliency of a pixel is represented by the color contrast of this pixel with the color of all other pixels in the image. To simulate the structure of the center-circle resistance of the receptive field of the human eye, we adopt the method of intralayer contrast for various attention mechanism features, that is, open a neighborhood window around each pixel, and divide this neighborhood. The window is regarded as the receptive field and the feature contrast between the current pixel of the genetic neural network and the rest of the pixels in the neighborhood window is taken as the significant value of the pixel at the current scale, it can be seen that the difference between the center and the periphery can best reflect the saliency of the image. After the attention map is obtained, there will be a situation where there are many contrast maxima for a certain feature, and a large number of significant peaks will appear at this time. If these feature attention maps with a large number of significant peaks are directly merged, other features with fewer significant peaks in Figure 4 will be suppressed, so they need to be normalized before merging the attention maps to generate a saliency map.

The article "Research on Image Segmentation Algorithm Based on Multimodal Hierarchical Attention Mechanism and Genetic Neural Network" was published in 2022. Journal: Comput Intell Neurosci.

The HxWxN matrix of the original multimodal hierarchy map, where *H* and *W* are height and width, respectively, and *N* is the number of images. These multimodal hierarchy maps capture the multimodal hierarchy map after projecting the multimodal hierarchy map onto the RGB image plane, but before filling in the missing multimodal hierarchy values. In addition, the multimodal hierarchy nonlinearity of the Kinect device has been removed, and the values of each multimodal hierarchy graph are in meters. The first module, called the initial resource recommendation module, uses a static model to directly and accurately build the relationship between resources and completion times. Therefore, the model can be used to provide cloud tenants with specific virtual machine configuration and quantity recommendations based on workload and deadline requirements of tenant genetic neural network tasks. The initial resource recommend module uses the regression model to construct the above relationship:

(11) $$\begin{array}{c} \left\{\begin{array}{c} W_{CONVER}^{I,I-1}\left(i-1,i\right)+W_{CONVER}^{I,I-1}\left(0,0\right)=1\\ W_{CONVER}^{I,I-1}\left(i-1,i\right)=CONVER\left[i,sig\mathrm{mod}\left(i\right)\right]. \end{array}\right. \end{array}$$

The initial multimodal level estimation part uses the monocular RGB image as input and uses the codec network structure to realize the initial rough estimation of the multimodal level of the scene, and narrow the scope for the subsequent multimodal level refinement. The multimodal hierarchy refinement part is based on the initial multimodal hierarchy results obtained above, combined with more accurate sparse multimodal hierarchy sampling, to further optimize the multimodal hierarchy results. The system was developed and implemented in Alibaba Cloud based on the Hadoop genetic neural network framework. The actual test of the system shows that (1) when determining the initial genetic neural network resource quantity, the prediction accuracy of the system's prediction model for the task completion time is 98.4%; (2) it is compatible with other existing resource management systems in the field. In contrast, the system can save up to 30.8% of the cost of renting genetic neural network resources for cloud tenants while ensuring that tasks are completed on time:

(12) $$\begin{array}{c} \sum_{y,k}^{y+k}\left(S\left(i|,|i|-|1\right)-S\left(i|-|1|,|i\right)\right)+\sum_{y,k}^{y+k}\left(W\left(i|,|i|-|1\right)-W_{CONVER}^{I,I-1}\left(i|-|1|,|i\right)\right)=0. \end{array}$$

The experiment collects the top c words with the highest word frequency from the question answering training pairs in the VQA dataset and removes useless stop words, and uses these c words as the attribute image segmentation node table of the experiment. Then the experiment builds a multilabel image dataset with the MSCOCO image caption dataset based on the attributes of this attribute image segmentation node table. The labels of the images in this dataset come from the words whose corresponding subtitles appear in the attribute image segmentation node table. The experiments train a multilabel image classifier as an attribute detector on this multilabel image dataset. The multilabel image classifier uses VGG-19 as the basic network structure and replaces the activation function and loss function of the last layer with the Sigmoid function and the SigmoidCrossEntropy function to achieve the task of multilabel classification. When the hole rate is *d* = 8, the features that can be extracted by the hole convolution are started at four positions (the 1st, 3rd, 5th, and 7th after the relative starting position). At this time, the data distribution of the sensed points at relative positions 5 and 7 can no longer reflect the original data characteristics.

The article "Research on Image Segmentation Algorithm Based on Multimodal Hierarchical Attention Mechanism and Genetic Neural Network" was published in 2022. Journal: Comput Intell Neurosci.

### 4.3. Image Segmentation Model Weight Replacement

Usually, the attention mechanism is regarded as a parameterizable attention mechanism, which weights the input to the next layer in a probabilistic way, so it is also differentiable. The parameterized soft attention mechanism can be embedded in the neural network to automatically learn attention features, and the gradient can be inherited from the neural network according to the gradient derivation method, and back-propagated to other parts of the neural network model. The feature attention distribution probability *i* represents the attention degree of the i-th feature vector when the query *q* of the related task is given. Next, we further summarize the feature vectors input to the neural network. Because the relationship between these features may be highly nonlinear, this relationship is difficult to observe directly. This module uses a neural network to build the prediction model of this part, because the neural network has a better ability to construct nonlinear relationships between features when the amount of training data is sufficient. In this module, the data used for training comes from the real-time running status features collected every 5 seconds during the running of the genetic neural network task, and each running task can generate hundreds or thousands of such features so that the neural network can get enough training data:

(13) $$\begin{array}{c} ℜ\left(i,\;\cos\;c\right)=\left[\begin{array}{ccc} f\left(i,\;\sin\;c\right) & i & 1\\ i & f\left(i-n,\;\sin\;c\right) & i\\ 1 & i & f\left(1,\;\sin\;c\right) \end{array}\right]. \end{array}$$

Due to the large scale of the network and the need for a lot of data training, we used NYU-Depth. The network is trained on the raw data in the v2 dataset. During the experiment, we use the official toolkit to preprocess these unprocessed raw data, including left and right view correction, noise removal, image cropping, etc. In the experiment, we strictly separate the test data and training data: the scene where the 654 pictures in the official test data set are located is removed from the original data, and the remaining data is sampled at even intervals to obtain 43k synchronized RGB. Multimodal hierarchical image pairs are used as training data for all experiments. The resolution of each training data is 427 × 561.

The article "Research on Image Segmentation Algorithm Based on Multimodal Hierarchical Attention Mechanism and Genetic Neural Network" was published in 2022. Journal: Comput Intell Neurosci.

The second module is called the elastic resource management module. The module in Figure 5 employs a multimodal neural network-based predictive model to adjust the amount of computing resources in real time. At the same time, this module can also use a series of expansion strategies to decide when to perform resource expansion operations and the number of resources that need to be increased. Features such as number of resources and task running settings (static features) can be used to predict task completion time well. The above multimodal features can be used to predict the completion time of genetic neural network tasks through neural networks. Another advantage of the multimodal neural network is that it can maximize the use of the deep information hidden in the above multimodal features, while reducing the “noise” generated when using different modal features. The neural network includes a neural network structure based on multimodal hierarchical Hotellin autoencoder for feature fusion and noise reduction. The structure in Table 2 is very suitable for learning the features of multiple modalities at the same time and maximizes the correlation between different modal features and reduces the interference between irrelevant features.

The article "Research on Image Segmentation Algorithm Based on Multimodal Hierarchical Attention Mechanism and Genetic Neural Network" was published in 2022. Journal: Comput Intell Neurosci.

After the tenant has given the workload and deadline of the genetic neural network task, the allocator in the initial resource recommendation module will provide the user with the most cost-effective resource allocation strategy to rent the genetic neural network resource on the public cloud. The initial resource recommendation module is an offline tool. During the establishment process, it is necessary to construct the relationship between the task workload, the amount of genetic neural network resources, and the completion time. To this end, the initial resource recommendation module adopts a regression model to obtain the above relationship. The initial resource recommendation module aims to provide users with initial resources that can complete the number of genetic neural networks just before the deadline, and this system does not recommend reducing genetic neural network resources during the genetic neural network process of the task. The main reason is that when the task starts running, deleting the virtual machine from the cloud genetic neural network cluster may cause the data loss of the completed genetic neural network, so that the part of the genetic neural network that has been completed starts the genetic neural network again.

## 5. Application and Analysis of Image Segmentation Model Based on Multimodal Hierarchical Attention Mechanism and Genetic Neural Network

### 5.1. Evaluation Criteria of Attention Mechanism

The channel domain attention mechanism is mainly reflected in the channel of the feature map. It takes the feature map as the unit and assigns different weight values to each channel, and the weight value is a vector. For each feature map C, the channel attention mechanism learns different attention weights in each channel dimension C, and has the same weight in the plane dimension W. The biggest difference is that the hard attention mechanism is nonparameterized and nondifferentiable. It selects one of the inputs directly to the next layer, that is, only pays attention to one position at a time. The soft attention mechanism will pay attention to all the data, and the genetic neural network will output the attention weight value of each data, and it is not limited by any constraints. The specific situation of the first multiscale convolutional layer when *M* = 3 is given, in which the smallest scale is completed by traditional convolution, that is, *d* = 1; when realizing the convolution kernel of mesoscale and large-scale receptive field, the void ratios *d* = 2 and *d* = 4 were used, respectively. During an iterative training, we no longer pay attention to these places that do not meet the screening constraints, that is, only select a certain area in the image, and then reset its weight to 1, and the weights of the areas in Figure 6 are all set to 0. Because the hard attention mechanism is a nondifferentiable attention mechanism, the training process of hard attention is usually trained using reinforcement learning.

The article "Research on Image Segmentation Algorithm Based on Multimodal Hierarchical Attention Mechanism and Genetic Neural Network" was published in 2022. Journal: Comput Intell Neurosci.

The task is decomposed into a global estimation network and a local estimation network, in order to take into account the multimodal level of the scene as a whole and details. However, this network structure design uses two fully connected layers in the global estimation network, which not only makes the network parameters too many but also reduces the prediction efficiency of the network. In the training process, the encoder extracts, encodes, and abstracts image features; while the decoder performs reverse conversion according to the compressed representation of the encoder to realize the conversion from the RGB image domain to the scene multimodal level domain. In addition, in order to enable the network to take into account global information and local details, we added short-circuit connections between the corresponding layers of the codec network to achieve information-sharing between the codec networks in Table 3, and obtain a more accurate multimodal hierarchical prediction results.

For the image model, experiments are carried out from ResNet. The last image segmentation layer of 152 extracts attention mechanism features. For a 448 × 448 image, the experiment results in a feature map of size 14 × 14 × 2048. Each 2048-dimensional feature of the feature map corresponds to a 32 × 32 area of the input image. In the experiment, the four-way 2D GRU is used instead of the two-way GRU to encode the context of the original feature map so that each region can perceive its surrounding area information. The dimension of the hidden state in the 2D GRU is set to be the same as the problem feature, which is 2400 dimensions. Therefore, after the experiment passes the original feature map to the 2D GRU module, the experiment obtains a 14 × 14 × 2400 context-aware feature map. Then the experiment maps the question features and the attention mechanism features known by the context of the image to the same 512-dimensional space, and then performs the attention mechanism attention operatio:

(14) $$\begin{array}{c} \exp\left[\log\left(f\left(i,j,k\right)\right)\right]+\exp\left[\log\left(g\left(i,j,k\right)\right)\right]+\exp\left[\log\left(z\left(i,j,k\right)\right)\right]=\log\left(f,g,z|i,j,k\right). \end{array}$$

The paper shows the network model of the attention mechanism module of the image segmentation block. It is assumed that after an image is input, some features are obtained after passing through some image segmentation layers, and then the CBAM module degenerates the neural network image at the channel level and the spatial level in turn. Finally, the learned attention features and the features after the previous image segmentation layer feature learning are multiplied between elements to achieve adaptive feature learning of significant discriminative features. The experiment assigns a weight score to each region to model the relationship between that region and the question currently being asked. Unlike the semantic attention mechanism, which measures the semantic similarity between the question and the attribute word through the dot product of two vectors, in the attention mechanism, the experiment multiplies the two vectors element by element and then sends it to the multilayer perceptron method to learn the association between the question and each image region.

The article "Research on Image Segmentation Algorithm Based on Multimodal Hierarchical Attention Mechanism and Genetic Neural Network" was published in 2022. Journal: Comput Intell Neurosci.

### 5.2. Image Segmentation Simulation Implementation of Genetic Neural Network

The Genetic Neural Network dataset contains real image data collected from urban, rural, and highway scenes, with up to 15 cars and 30 pedestrians in each image, with varying degrees of occlusion and truncation. The entire dataset includes 389 pairs of stereo images and optical flow maps, 39.2 of attention-mechanism ranging sequences, and over 200 k images of 3D annotated objects. The images are sampled and synchronized at 10 Hz. The experiment proposes to replace the traditional bidirectional recurrent neural network model with a two-dimensional recurrent neural network to encode the context information of the image region and to effectively learn the dependencies between regions from two dimensions and four directions. Experiments show that the 2D image segmentation neural network can outperform the original bidirectional image segmentation neural network and achieve significant improvement over the attention model that does not use context encoding. In addition, this chapter also conducts more experiments on VQA v2.0 on a more balanced attention mechanism question answering dataset, and more extensive ablation experiments are also implemented and studied.

(15) $$\begin{array}{c} \text{softmax}\left(z\left(p,q\right)\right)-\text{softmax}\left(z\left(p-1,q-1\right)\right)-\ldots -\text{softmax}\left(z\left(1,1\right)\right)=\text{max}\left(p,q\right). \end{array}$$

After the genetic neural network task starts running, the monitors in the elastic resource management module will continuously (every 5 seconds) collect data about the task running status and virtual machine resource utilization from the genetic neural network cluster. These raw data are preprocessed and sent to the predictor. The predictor will continuously use these data to predict the completion time of the task and provide necessary elastic resource expansion operations when it is predicted that the task cannot be completed before the deadline. Specifically, the first two layers of convolution kernels in the original FCN are split into multiple groups, in which the larger-scale part is realized by whole convolution, and the smaller-scale part is realized by ordinary convolution. These characteristics include computing resource characteristics, task processing speed characteristics, and resource utilization characteristics. Among them, the task processing speed and resource utilization characteristics in Figure 7 are time series characteristics, while the genetic neural network resource characteristics are nontime series characteristics.

The article "Research on Image Segmentation Algorithm Based on Multimodal Hierarchical Attention Mechanism and Genetic Neural Network" was published in 2022. Journal: Comput Intell Neurosci.

However, the 2D GRU has two update gates and two reset gates, which control the flow of information in two vertical dimensions, respectively. Specifically, the experiments use a pretrained image segmentation neural network model to extract the attention mechanism features of local regions. In the experiment, the feature map of the last image segmentation layer of the image segmentation neural network model is expressed as the initial attention mechanism of the experiment, which can retain the complete spatial information of each region. This part of the network structure takes single-purpose RGB images as input and uses the powerful scene understanding and function fitting capabilities of multimodal hierarchical neural networks to perform relatively multimodal hierarchical predictions on the surface structure of objects:

(16) $$\begin{array}{c} \frac{\Delta mv+\Delta m\left(v,v\left(t\right)\right)+\Delta m\left(v,v\left(x,y\right)\right)}{\Delta m\left(v,v\prime \right)-\Delta mv}=1. \end{array}$$

The error-prone regions of the mechanism method (weak multimodal hierarchy, presence of illumination differences, etc.) can obtain more robust multimodal hierarchy estimation results. The design of the generative network part adopts the design idea similar to that of the multimodal level initialization part, and also adopts U-Net, which contains an encoding network and a decoding network. The encoding network consists of a series of concatenated image segmentation modules to compress the input information and obtain a feature-encoded representation of the input. Since the receptive field of the network is very important in the pixel-level estimation task, two concatenated image segmentation layers are used in the connected part of the encoder-decoder network to further expand the network receptive field.

### 5.3. Example Application and Analysis

That is, the number of neurons can be adjusted between 8, 64, and 128 according to the complexity of the temporal features in the specific data and the training ability of the model. In order to maintain the robustness of this part, the pruning operation is added, and its dropout rate is set to 0.8. The frame rate of all data is 30 Hz, and the sensor resolution is 640 × 480. The moving trajectory of the sensor is obtained by a high-precision motion capture system and eight high-speed tracking cameras (100 Hz). In addition, this dataset provides accelerometer data from Kinect and provides an evaluation criterion to measure the quality of the estimated camera trajectory of the attention mechanism SLAM system. In order to better construct the mapping relationship ƒ, the Pearson correlation coefficient is first used in this module to explore the linear correlation between these features and completion time. Among them, the Pearson correlation coefficient is usually used to describe the linear correlation between two variables, and its value is the product of the covariance of the two variables divided by their standard deviations. The Pearson correlation coefficient takes values between –1 and 1, where 1 is a perfectly positive linear correlation, 0 is no linear correlation, and –1 is a perfectly negative linear correlation. Through the Pearson correlation coefficient between each feature of the genetic neural network and the completion time, we can know the importance of these features to the prediction results when making predictions. Specifically, a feature with a larger linear correlation indicates that it will also have a larger impact on completion time:

(17) $$\begin{array}{c} \left\{\begin{array}{c} \text{sin}h\left(x,t\right)-h\times \text{sin}h\left(x-1,t\right)=h\left(x,t\right)\\ \text{tan}h\left(x,t\right)-k\times \text{tan}h\left(x-1,t\right)=k\left(x,t\right) \end{array}.\right. \end{array}$$

The key of genetic neural network image segmentation is to extract more rich discriminative features of the image, while the current genetic neural network image segmentation methods can only learn particularly significant discriminative features but cannot learn secondary significant discriminative features. For two species that are particularly similar between classes, it is often impossible to distinguish the category of the current species by only relying on the main salient discriminative features of the two extracted. The method based on the adversarial complementary attention mechanism proposed in this paper can learn relatively minor and significant discriminative features, which solve the problem that the current genetic neural network image segmentation method can only learn the main and significant discriminative features and improve the genetic neural network. The improved algorithm adopts a new spatial transformation method and uses the statistical characteristics of the image to inherit the mean information of the neural network image, so as to obtain a clearer saliency map. Then, through the minimum circumscribed rectangle of the salient region of the genetic neural network, new processed images are correspondingly cut out from the original input Figure 8, and finally these new processed images are applied to the processing work of representative image selection, with fewer operations to get a more comprehensive representative image.

The article "Research on Image Segmentation Algorithm Based on Multimodal Hierarchical Attention Mechanism and Genetic Neural Network" was published in 2022. Journal: Comput Intell Neurosci.

For each attribute, the experiment trains an image segmentation neural network-based segmentation device, then the activation value of the semantic output layer of the image segmentation neural network constitutes the high-level semantic representation of the input image. Third, the knowledge attention module extracts knowledge that is helpful for answering specific questions by connecting the attributes detected in the image and external knowledge bases (such as Wikipedia). Simple connection methods such as addition or cascade cannot fully capture the complex relationship between features, so a feature fusion mechanism of high-order statistical representation is designed. Fourth, the joint learning module uses an elementwise multiplication method to fuse features from local regions, attributes, knowledge, and question, and then integrates into a softmax layer to predict the most likely answer:

(18) $$\begin{array}{c} \sin\left(\frac{\exp\left(x/t\right)+\exp\left(-x/t\right)}{\exp\left(x/t\right)-\exp\left(-x/t\right)}\right)+\cos\left\{\frac{\exp\left(x/t\right)+\exp\left(-x/t\right)}{\exp\left(x/t\right)-\exp\left(-x/t\right)}\right\}=1. \end{array}$$

This experiment will consider the quantitative relationship between these two features and completion time separately and plot it as an image. As shown in the paper, the total workload *w* of pending tasks is inversely proportional to the completion time, and the number of virtual machines *n* used for the genetic neural network is positively linearly related to the completion time. The other features used in this model can be considered to be linearly related to each other and do not interfere with each other. Therefore, the functional relationship to be fitted in the prediction model can be finally obtained. VQA is a large-scale attention mechanism question answering dataset, which contains 204,721 real pictures from COCO dataset and a scene picture containing 50,000 newly created abstract scene datasets. Experiments only evaluate experimental models on real images. For each image in the VQA dataset, three questions are annotated, and each question has 10 answers annotated from 10 different annotators.

The article "Research on Image Segmentation Algorithm Based on Multimodal Hierarchical Attention Mechanism and Genetic Neural Network" was published in 2022. Journal: Comput Intell Neurosci.

The experiments report the experimental results on two different tasks, namely the open attention mechanism question-answering task and the multiple choice attention mechanism question-answering task. In the open-ended task, the experiment selects the answer candidate with the largest activation value from all possible outputs as the answer, while in the polynomial task, the experiment selects only the answer with the largest activation value from the given candidates. Experiments collect the 3000 most frequently occurring answers in the training set as a general set of candidate answers. The experiment not only evaluates the experimental method on the validation set but also uses the test server to evaluate the experimental method on the test set.

## 6. Conclusion

Based on the multilevel modal attention mechanism, this paper proposes an improved image segmentation algorithm. First, the multisource multilevel attention network introduces an external knowledge base, and simultaneously uses the multisource information from the attention mechanism and knowledge to make the attention mechanism question-answering system for knowledge-based reasoning. The structure of GRU models the relationship between the upper, lower, left, and right dimensions of the image and four directions, which is more in line with the structural characteristics of the image. Finally, we achieve significantly better results than multilevel attention networks on the two largest VQA datasets. The design of the overall network adopts the idea from coarse to fine. Among them, the initial multimodal level rough estimation part draws on the existing CNN-based monocular multimodal level prediction method, uses the powerful scene understanding ability of the CNN network, and obtains a multimodal level of the scene from a single RGB image input. Then, the multimodal level refinement part optimizes the scene multimodal level on the basis of the obtained rough initial multimodal level, combined with sparse and accurate multimodal level sampling and RGB input, so as to obtain a more accurate multimodal level. In the multimodal level refinement part, we use a combination of adversarial loss, reconstruction loss, and smoothing loss to obtain more refined scene multimodal level recovery results and better model generalization ability. In this paper, we mainly extract the discriminative features between different layers at the same scale after using the adversarial complementary attention mechanism to extract the high-level discriminative features of the image and then divide the discriminative features of these different layers into two bilinear pooling is performed between the two, that is, the discriminative features between different layers are fused to enhance the representation ability of the image to improve the image segmentation ability of the genetic neural network under weak supervision. The experimental results show that compared with the existing algorithms based on deep convolutional neural networks, the method has a significant improvement in the quality of high-frequency detail reconstruction, and can obtain better visual effects and faster convergence speed.

The article "Research on Image Segmentation Algorithm Based on Multimodal Hierarchical Attention Mechanism and Genetic Neural Network" was published in 2022. Journal: Comput Intell Neurosci.

## Figures and Tables

**Figure 1:** Image neural network node topology.

**Figure 2:** Input polar coordinate distribution of original image sequence.

**Figure 3:** Saliency detection results of multimodal hierarchical images.

**Figure 4:** The distribution of the numerical fitting of the output of the genetic neural network.

**Figure 5:** Multimodal neural network image segmentation weight distribution.

**Figure 6:** Constraint hierarchy of genetic neural network.

**Figure 7:** Task utilization of genetic neural network cluster.

**Figure 8:** Neural network image segmentation mean Information distribution.

**Table 1:** Properties of biological attention mechanism.

Unit case	Mean square error	Confidence value	Covariance value
Biological attention	0.061	1.917	0.326
Discriminative features	0.064	1.881	0.357
Suppress responses	0.067	1.845	0.388
Secondary salient	0.070	1.809	0.419
Unconventional features	0.072	1.773	0.45
Attention mechanism	0.075	1.737	0.481

**Table 2:** Multimodal hierarchy distributed autoencoder description.

The neural network including content			Multimodal hierarchy distribution		
Tasks	Reduction	Modalities	Tasks	Reduction	Modalities
0.084	0.979	0.064	0.367	0.169	0.223
0.782	0.205	0.355	0.324	0.318	0.141
0.085	0.157	0.688	0.191	0.884	0.526
0.904	0.272	0.790	0.998	0.970	0.721
0.334	0.502	0.144	0.296	0.398	0.131

**Table 3:** Information sharing of codec networks.

Information code number	Accurate multimodal hierarchical prediction text
Fuse the information of *x* − 1	Time (time_t^*∗*^)NULL);
Confidence level *k*(*t*)	Srandom((unsigned int)
Adjusts the information sin*h*(*x* − 1)	Int value = (arc4random() % *x*) + 1;
The multi-modal body of evidence *r*!	-(int)getrandomnumber:
Adjustment factor for *x*/*t*	Int value = (arc4random() % *x*) + 1;
According to equations (*n* − *r*)!	(int)from to:(int) to case)
The selected mode Δ*mv*	Return (int) (from +)
Make decisions according to *f*(*i*, *j*)	(arc4random() % (to – from + 1)));
Find the continuous interval Δ*m*(*v*, *v*′)	Int *x* = arc4random() % 100;
With the highest accuracy *f*(*i*, *j*, *k*)	Int value = arc4random() % *x*;

The article "Research on Image Segmentation Algorithm Based on Multimodal Hierarchical Attention Mechanism and Genetic Neural Network" was published in 2022. Journal: Comput Intell Neurosci.

## Data Availability

The data used to support the findings of this study are available from the corresponding author upon request.
